# Microvascular resistance reserve in the presence of functionally significant epicardial stenosis and changes after revascularization

**DOI:** 10.14814/phy2.15627

**Published:** 2023-03-10

**Authors:** Yoshihiro Hanyu, Masahiro Hoshino, Eisuke Usui, Tomoyo Sugiyama, Yoshihisa Kanaji, Masahiro Hada, Tatsuhiro Nagamine, Kai Nogami, Hiroki Ueno, Kodai Sayama, Kazuki Matsuda, Tatsuya Sakamoto, Taishi Yonetsu, Tetsuo Sasano, Tsunekazu Kakuta

**Affiliations:** ^1^ Division of Cardiovascular Medicine Tsuchiura Kyodo General Hospital Ibaraki Japan; ^2^ Department of Interventional Cardiology Tokyo Medical and Dental University Tokyo Japan; ^3^ Department of Cardiovascular Medicine Tokyo Medical and Dental University Tokyo Japan

**Keywords:** chronic coronary syndrome, coronary flow reserve, fractional flow reserve, microvascular resistance reserve, percutaneous coronary intervention

## Abstract

In the presence of functionally significant epicardial lesions, microvascular resistance reserve (MRR) calculation needs incorporation of collateral flow. Coronary fractional flow reserve (FFR_*cor*_) requiring coronary wedge pressure (P_*w*_), which is an essential part of the true MRR calculation, is reportedly estimated by myocardial FFR (FFR_*myo*_) not requiring P_*w*_ measurement. We sought to find an equation to calculate MRR without the need for P_*w*_. Furthermore, we assessed changes in MRR after percutaneous coronary intervention (PCI). An equation to estimate FFR_*cor*_ was developed from a cohort of 230 patients who underwent physiological measurements and PCI. Corrected MRR was calculated using this equation and compared with true MRR in 115 patients of the different set of the validation cohort. True MRR was calculated using FFR_*cor*_. FFR_*cor*_ and FFR_*myo*_ showed a strong linear relationship (*r* ^2^ = 0.86) and an equation was FFR_*cor*_ = 1.36 × FFR_*myo*_ – 0.34. This equation provided no significant difference between corrected MRR and true MRR in the validation cohort. Pre‐PCI lower coronary flow reserve and higher index of microcirculatory resistance were independent predictors of pre‐PCI decreased true MRR. True MRR significantly decreased after PCI. In conclusion, MRR can be accurately corrected using an equation for FFR_*cor*_ estimation without P_*w*_.

## Graphical abstract

Corrected MRR was calculated using measured MRR (MRRapp) and estimated FFRcor by the equation: corrected MRR = MRRapp × (FFRmyo/FFRcor) = MRRapp × FFRmyo/(1.36 × FFRmyo−0.34). There is no significant difference between true MRR and corrected MRR in the validation cohort.

## 1 INTRODUCTION

Microvascular dysfunction has been increasingly acknowledged as a relevant cause of myocardial ischemia. (Camici et al., 2015; Camici & Crea, 2007; Crea et al., 2014) Nonetheless, limited practical tools are available to quantify coronary microvascular function, particularly in the presence of significant epicardial coronary artery stenosis. (Fearon et al., 2003; Kelshiker et al., 2022; Layland et al., 2013; Travieso et al., 2022). Recently, microvascular resistance reserve (MRR), as an index specific for the assessment of microcirculation, has been proposed. (de Bruyne et al., 2021) MRR has been reported to be independent of autoregulation and myocardial mass and an operator‐independent measure of the absolute value of microvascular resistance reserve. (de Bruyne et al., 2021) The theoretical framework of MRR and its derivation by physiological measures have been presented. The authors indicated that MRR should be corrected in the presence of significant epicardial stenosis as described for the index of microcirculatory resistance (IMR) correction by Aarnoudse et al. and Yong et al. (Aarnoudse et al., 2004; Fearon et al., 2013) Epicardial stenosis and microvascular dysfunction may coexist. (Taqueti & Di Carli, 2018) Identification or discrimination of these factors relevant to myocardial ischemia is challenging but might contribute to tailored management and therapeutic strategy for patients with chronic coronary syndrome. Thus, we sought to derive the equation of linear regression from estimating coronary fractional flow reserve (FFR_*cor*_) in the derivation cohort and to validate the derived method for corrected MRR values using calculated FFR_*cor*_ and apparent value of MRR (MRR_*app*_) in the different set of the validation cohort. We then compared these corrected MRR values with those corrected using Yong's equation, (Yong et al., 2013) if Yong's equation is valid for the correction of MRR. We also assessed the changes in MRR after percutaneous coronary intervention (PCI) in the combined study population of derivation and validation. We further evaluated pre‐PCI cut‐off values of true MRR corresponding to coronary flow reserve (CFR), IMR, and resistive reserve ratio (RRR) threshold values. Predictive factors for pre‐PCI low true MRR values were also evaluated.

## 2 METHODS

### 2.1 Study design and patient population

The derivation cohort was chosen from our institutional PCI database (Figure 1). The age and sex‐matched validation cohort was also identified from this database in the same fashion described below. The present analysis was performed in a post hoc manner. Two hundred and thirty patients of the derivation cohort were randomly chosen from the all‐comers institutional elective PCI registry database enrolling our regular clinical population according to the following inclusion criteria: age >20 years old with chronic coronary syndrome and the detection of an identifiable, single de novo culprit lesion located in the proximal portion of a native coronary artery and symptomatic ischemia or objective ischemia according to non‐invasive stress testing and/or fractional flow reserve (FFR) measurements. Exclusion criteria included angiographically significant left main disease, renal insufficiency with baseline serum creatinine level >1.5 mg/dL, cardiomyopathy, and congestive heart failure. All patients underwent FFR‐guided PCI and pre‐ and post‐PCI physiological assessments with accessible data quality. After PCI, we further excluded patients with periprocedural myocardial infarction as defined by the Fourth Universal Definition of Myocardial Infarction, (Thygesen et al., 2018) based on a blood sample taken an average of 20–24 h, symptoms, and other objective findings after PCI completion, because such events have been reported to affect post‐PCI physiological measurements. (Silvain et al., 2021) Patients with minor cardiac troponin elevation, without other manifestations required by definition mentioned above, were included in the final analysis. The age and sex‐matched validation cohort of 115 patients was similarly identified from the institutional registry. A representative case undergoing FFR‐guided PCI with pre‐ and post‐PCI angiograms and physiological data are shown in Figure 2. This study was conducted in compliance with the institutional ethics committee guidelines and received its approval (TKGH #2022FY83). The present study also complied with the Declaration of Helsinki for the investigation of human beings, and all patients provided written informed consent before the institutional registry enrollment for future investigations. Prompt optimal medical therapy was initiated in all patients before PCI.

**FIGURE 1:** Study flow chart. Abbreviations: CABG, coronary artery bypass grafting; CCS, chronic coronary syndrome; PCI, percutaneous coronary intervention.

**FIGURE 2:** Representative case with CCS who underwent FFR‐guided PCI with pre‐ and post‐PCI physiological evaluations. A 70‐year‐old man with CCS underwent FFR‐guided second‐generation drug‐eluting stent implantation in the right coronary artery with pre‐ and post‐intervention physiological evaluations. Abbreviations: CFR, coronary flow reserve; FFR, fractional flow reserve; FFR_*cor*_, coronary fractional flow reserve; FFR_*myo*_, myocardial fractional flow reserve; IMR, index of microcirculatory resistance; MRR, microvascular resistance reserve; PCI, percutaneous coronary intervention; RRR, resistive reserve ratio. Other abbreviations are shown in Figure 1.

### 2.2 Pre‐ and post‐PCI physiological measurements and analysis

Coronary angiography and PCI procedure were performed by standard techniques. Coronary angiograms were analyzed quantitatively using a CMS‐MEDIS system (Medis Medical Imaging Systems). The PCI techniques and imaging devices, such as intravascular ultrasound or optical coherence tomography, and stent type (drug‐eluting stent) were at the interventionalists' discretion. Pre‐ and post‐PCI FFR, CFR, and IMR measurements were performed, as previously described. (de Bruyne et al., 2001; Fearon et al., 2003; Matsuda et al., 2016; Pijls et al., 1996) Briefly, coronary physiological measurements were obtained by a 6F guiding catheter via radial approach using a pressure–temperature sensor guidewire and analyzing systems (PressureWire X Guidewire, Abbott Laboratories, Il, USA, RadiAnalyzer, St, Jude Medical, St Paul, Minnesota, UAS and CoroFlow, Coroventis Research AB, Uppsala, Sweden). After the administration of a bolus of intracoronary nitrate (200 μg), the wire sensor was advanced and positioned as far distally in the target vessel as practical. Hyperemia was induced by infusion of adenosine or adenosine triphosphate into an antecubital vein at a rate of 140 μg/kg/min or 160 μg/kg/min, respectively. FFR was calculated as the ratio of distal coronary pressure to proximal pressure at stable hyperemia. CFR was obtained using the thermodilution method as the ratio of resting transit time divided by hyperemic transit time (T_*mn*_). IMR was calculated as the distal coronary pressure at maximal hyperemia divided by the inverse of the hyperemic T_*mn*_. RRR was calculated by CFR adjusted using the ratio between resting and hyperemic distal coronary pressure. (Lee et al., 2020) The P_*a*_, P_*d*_, and P_*w*_ were recorded during balloon dilatation during PCI. Post‐PCI physiological measurements were also performed in a similar manner after post‐stenting high‐pressure dilatation using a noncompliant balloon and/or additional stenting guided by physiological and intravascular imaging at the operators' discretion and when the operator considered as final as the PCI procedure.

### 2.3 Formula derivation and MRR correction

As reported in the study by Yong et al., the regression formula between FFR_*cor*_ and FFR_*myo*_ of best fit by a straight line was obtained in the derivation cohort. This formula was tested in the validation cohort. MRR is defined as the ratio of true resting to hyperemic microvascular resistance (R_*μ*_), as recently described. (de Bruyne et al., 2021) The theoretical framework of calculating resting R_*μ*_, hyperemic R_*μ*_, MRR, and the relationship between FFR, CFR, and MRR was shown by de Bruyne et al. (2021) Briefly, MRR is defined by the following equation:

$$\begin{array}{c} \begin{array}{c} \mathrm{MRR}=\text{resting}\;R_{\mu }\;/\;\text{hyperemic}\;R_{\mu }\;=\;P_{a,\;\text{rest}}\;/\;Q_{\text{rest}}\;÷\;P_{d,\;\text{hyper}}/\;Q_{\max}\\ \;=\left(Q_{\max}\;/\;Q_{\text{rest}}\right)\;\times \;\left(P_{a,\;\text{rest}}\;/\;P_{d,\;\text{hyper}}\right) \end{array} \end{array}$$

where P_*a, rest*_ and P_*d*, *hyper*_ are resting aortic and hyperemic distal coronary pressure, respectively, and Q_*rest*_ and Q_*max*_ are the resting and hyperemic absolute coronary blood flow. This equation can also be described using CFR and FFR by the following equation:

$$\mathrm{MRR}=\left(\mathrm{CFR}\;/\;\mathrm{FFR}\right)\;\times \;\left(P_{a,\;\text{rest}}/P_{a,\;\text{hyper}}\right)$$

where FFR indicates FFR_*myo*_. As suggested by De Bruyne et al., true MRR, in the presence of significant epicardial stenosis, should be derived by correcting MRR_*app*_ and can be expressed by the following:

$$\begin{array}{c} \text{True}\;\mathrm{MRR}=\mathrm{CFR}\;/\;{\mathrm{FFR}}_{\mathrm{cor}}\;\times \;\left(P_{a,\;\text{rest}}\;/\;P_{a,\;\text{hyper}}\right)\\ \;={\mathrm{MRR}}_{\mathrm{app}}\;\times \;\left({\mathrm{FFR}}_{\mathrm{myo}}\;/\;{\mathrm{FFR}}_{\mathrm{cor}}\right) \end{array}$$

where true MRR and MRR_*app*_ represent corrected MRR and measured MRR, respectively. Consequently, using the formula of the relationship between FFR_*myo*_ and FFR_*cor*_, we can obtain a corrected MRR. In the validation cohort, we also compared true MRR values with corrected MRR values using Yong's equation (Yong et al., 2013) if there is no statistically significant difference between these two values obtained by each of the two equations for FFR_*cor*_ estimation. We summarized definitions of all physiological parameters below. We further assessed the changes in MRR values in the total cohort, including both derivation and validation cohorts (345 patients) after PCI.

CFR = Q_*max*_ / Q_*rest*_ ≈ T_*mn, rest*_ / T_*mn*, *hyper*_

Calculated FFR_*cor*_ = 1.36 × FFR_*myo*_ – 0.34

Measured FFR_*cor*_ = FFR_*cor*_ = (P_*d, hyper*_ − P_*w*_) / (P_*a, hyper*_ − P_*w*_)

IMR_*rest*_ = (P_*d, rest*_ – P_*v*_) / Q_*rest*_ ≈ P_*d, rest*_ × T_*mn, rest*_

IMR_*hyper*_ = (P_d*, hyper*_ – P_v_) / Q_*max*_ ≈ P_*d, hyper*_ × T_*mn*, *hyper*_

IMR = Corrected IMR = P_*a, hyper*_ × T_*mn*, *hyper*_ × (P_*d, hyper*_ − P_*w*_) / (P_*a, hyper*_ − P_*w*_)

MRR_*app*_ = Measured MRR

= CFR × (P_*a, rest*_ / P_*d, hyper*_)

= (CFR / FFR_*myo*_) × (P_*a, rest*_ / P_*a, hyper*_)

Corrected MRR = CFR / (1.36 × FFR_*myo*_ − 0.34) × (P_*a, rest*_ / P_*a, hyper*_)

Corrected MRR by Yong's formula = CFR / (1.34 × FFR_*myo*_ − 0.32) × (P_*a, rest*_ / P_*a, hyper*_)

True MRR = (CFR / FFR_*cor*_) × (P_*a, rest*_ / P_*a, hyper*_)

RRR = IMR_*rest*_ / IMR_*hyper*_

P_*a*_ = aortic pressure (mmHg)

P_*a, rest*_ = aortic pressure under resting conditions

P_*a, hyper*_ = aortic pressure at maximum hyperemia

P_*d*_ = distal coronary pressure (mmHg)

P_*d, rest*_ = distal coronary pressure under resting conditions

P_*d, hyper*_ = distal coronary pressure at maximum hyperemia

P_*v*_ = mean right atrial pressure (mmHg)

Q = coronary blood flow (ml/min)

Q_*rest*_ = coronary blood flow under resting conditions

Q_*max*_ = maximum coronary blood flow at maximum hyperemia

R_*μ*_ = microvascular resistance (WU)

R_*μ, rest*_ = microvascular resistance under resting conditions

R_*μ, hyper*_ = microvascular resistance at maximum hyperemia

T_*mn*_ = mean transit time (s)

T_*mn, rest*_ = mean transit time under resting conditions

T_*mn*, *hyper*_ = mean transit time at maximum hyperemia

### 2.4 Statistical analysis

Statistical analyses were performed using R version 4.0.3 (The R Foundation for Statistical Computing) and SPSS version 25.0 (IBM Corporation). Categorical data were expressed as numbers and percentages and compared by the chi‐square or Fisher's exact tests. Continuous data were expressed as median (interquartile range) and analyzed using the Mann–Whitney *U* test. Paired *t*‐tests were used to compare the different methods for FFR and MRR values. Pearson's correlation analyses were used to evaluate the relationship between variables. Bland–Altman analyses we applied to test for agreement. The kappa statistic was used to test the interrater reliability of MRR values before and after PCI. Receiver operating characteristic curves were analyzed to assess the best cut‐off values of pre‐PCI true MRR corresponding to the CFR, IMR, and RRR cut‐off values, respectively. The optimal cut‐off value was determined by the Youden index. Univariable and multivariable logistic regression analyses were performed to predict pre‐PCI decreased true MRR. A value of *p* < 0.05 was considered statistically significant.

## 3 RESULTS

### 3.1 Baseline patient characteristics, angiographical, and physiological findings

Baseline patients' characteristics, angiographic, and physiological data in the derivation and validation cohorts are shown in Table 1. The median age of the total study population was 70 (63–75), and 85.0% were men. No significant differences in coronary risk factors are observed between the derivation and validation cohorts. The median pre‐PCI FFR and CFR were 0.71 and 1.97, respectively. The median post‐PCI FFR and CFR were 0.87 and 2.52, respectively. No significant differences in pre‐PCI and post‐PCI physiological indices are observed between the derivation and validation cohorts.

**TABLE 1:** Patients' clinical, angiographic, and physiological characteristics.

	Overall (*N* = 345)	Derivation cohort (*N* = 230)	Validation cohort (*N* = 115)	*p* value
**Baseline characteristics**				
Age	70 (63–75)	71 (63–75)	70 (63–76)	0.38
Male	293 (84.9)	200 (87.0)	93 (80.8)	0.15
BMI	24.7 (22.4–26.7)	24.7 (22.5–26.6)	24.5 (26.9)	1.00
Hypertension	262 (75.9)	180 (78.2)	82 (71.3)	0.19
Diabetes mellitus	155 (44.9)	108 (46.9)	47 (40.8)	0.30
Dyslipidemia	193 (55.9)	126 (54.8)	67 (58.2)	0.57
Family history	52 (15.1)	32 (13.9)	19 (16.5)	0.52
LDL‐cholesterol	84 (65–107)	84 (64–106)	86 (67–115)	0.44
Smoking	224 (64.9)	150 (65.2)	74 (64.3)	0.91
eGFR	65.9 (51.8–78.3)	66.5 (52.8–77.8)	65.4 (51.8–81.1)	0.92
LVEF	63 (54–68)	63 (54–69)	62 (55–67)	0.44
SYNTAX score (pre‐PCI, per pts)	9 (5–14)	8 (5–13)	9 (5.5–14.5)	0.17
**Angiographical data (pre‐PCI)**				
Target vessel (RCA/LAD/LCX)	65/204/76 (19/59/22)	43/138/49 (19/60/21)	22/66/27 (19/57/24)	0.85
Lesion length	10.0 (7.2–13.9)	9.9 (7.1–13.6)	10.4 (7.5–14.2)	0.24
Diameter stenosis	58.8 (49.3–67.6)	58.6 (50.1–67.6)	59.5 (48.7–67.3)	0.99
Reference diameter	2.5 (2.2–2.9)	2.5 (2.2–2.9)	2.5 (2.2–2.9)	0.89
Minimum lumen diameter	1.0 (0.8–1.3)	1.0 (0.8–1.3)	1.0 (0.8–1.3)	0.94
**Physiological indices**				
Pre‐PCI FFR	0.71 (0.63–0.76)	0.71 (0.63–0.76)	0.70 (0.64–0.76)	0.70
Pre‐PCI CFR	1.97 (1.37–2.75)	1.96 (1.35–2.70)	2.0 (1.40–2.87)	0.96
Pre‐PCI IMR	20.2 (14.8–30.2)	20.4 (15.0–30.1)	19.5 (14.4–32.1)	0.62
T_*mn*_ at rest (pre‐PCI)	0.89 (0.57–1.25)	0.89 (0.57–1.28)	0.91 (0.56–1.16)	0.59
T_*mn*_ at hyperemia (pre‐PCI)	0.42 (0.29–0.65)	0.44 (0.28–0.63)	0.41 (0.29–0.80)	0.86
Post‐PCI FFR	0.87 (0.82–0.92)	0.87 (0.82–0.92)	0.87 (0.82–0.92)	0.89
Post‐PCI CFR	2.52 (1.7–3.42)	2.53 (1.70–3.44)	2.43 (1.72–3.40)	0.91
Post‐PCI IMR	19.6 (13.7–28.5)	20.1 (14.8–27.3)	19.2 (13.0–29.4)	0.36
T_*mn*_ at rest (post‐PCI)	0.71 (0.46–1.04)	0.72 (0.48–1.05)	0.66 (0.46–1.02)	0.51
T_*mn*_ at hyperemia (post‐PCI)	0.28 (0.20–0.40)	0.28 (0.21–0.40)	0.26 (0.19–0.44)	0.43

*Note*: Values are *n* (%) or median (first quartile, third quartile). Abbreviations: BMI, body mass index; CFR, coronary flow reserve; eGFR, estimated glomerular filtration rate; FFR, fractional flow reserve; IMR, index of microcirculatory resistance; LAD, left anterior descending artery; LCX, left circumflex artery; LDL, low‐density lipoprotein; LVEF, left ventricular ejection fraction; PCI, percutaneous coronary intervention; RCA, right coronary artery; T_*mn*_, mean transit time.

Abbreviations: BMI, body mass index; CFR, coronary flow reserve; eGFR, estimated glomerular filtration rate; FFR, fractional flow reserve; IMR, index of microcirculatory resistance; LAD, left anterior descending artery; LCX, left circumflex artery; LDL, low‐density lipoprotein; LVEF, left ventricular ejection fraction; PCI, percutaneous coronary intervention; RCA, right coronary artery; T_*mn*_, mean transit time.

### 3.2 Derivation of the equation for FFR_cor_ using FFR_myo_ , and its validation

The formula to estimate FFR_*cor*_ using FFR_*myo*_ in the derivation cohort was obtained as follows:

$${\mathrm{FFR}}_{\mathrm{cor}}=1.36\times {\mathrm{FFR}}_{\mathrm{myo}}-0.34\;\left(r^{2}=0.86,p<0.001\right)$$

when (Figure 3) this equation was applied in the validation cohort, no significant difference was detected between measured and calculated FFR_*cor*_ (0.59 ± 0.14 vs. 0.59 ± 0.13, *p* = 0.661; Figure 4a), and good correlation was observed between these two variables (*r* ^2^ = 0.90, *p* < 0.001; Figure 4b,c).

**FIGURE 3:** Derivation of the method to Calculate FFR_*cor*_. Linear regression analysis of measured FFR_*cor*_ versus FFR_*myo*_ in the derivation Cohort. Abbreviations are shown in Figure 2.

**FIGURE 4:** Validation of the method to calculate FFR_*cor*_. (a). Comparison between measured FFR_*cor*_ and calculated FFR_*cor*_. No significant difference was detected between the measured FFR_*cor*_ and the calculated FFR_*cor*_. (b). Linear regression of measured FFR_*cor*_ versus calculated FFR_*cor*_. (c). Corresponding Bland–Altman plot. The Red line denotes the bias of the agreement, and the green lines represent standard deviations of the bias. Abbreviations are shown in Figure 2.

### 3.3 Corrected MRR calculation using the above equation and comparison with true MRR values and those corrected by Yong's equation

Corrected MRR was calculated using measured MRR (MRR_*app*_) and calculated FFR_*cor*_ by the above‐described equation: MRR_*app*_ × (FFR_*myo*_ / FFR_*cor*_), where FFR_*cor*_ = 1.36 × FFR_*myo*_ − 0.34. No significant difference between true MRR and corrected MRR (4.13 ± 1.71 vs. 4.04 ± 1.53, *p* = 0.187) was detected (Figure 5a). There was also a good correlation and agreement between these two variables (Figure 5b,c). As seen from the equation for FFR_*cor*_ calculation, this equation is no more valid when FFR_*myo*_ is equal to or less than 0.25 since the denominator is close to zero or a negative number. Corrected MRR was significantly higher than MRR_*app*_ (4.04 ± 1.53 vs. 3.42 ± 1.35, *p* < 0.001).

**FIGURE 5:** Validation of the method to correct MRR. (a). Comparison between measured true MRR and corrected MRR. No significant difference was observed between true MRR and corrected MRR. (b). Linear regression of true MRR versus corrected MRR. (c). Corresponding Bland–Altman plot. The Red line denotes the bias of the agreement, and the green lines represent standard deviations of the bias. Abbreviations are shown in Figure 2.

When MRR_*app*_ was corrected using Yong's equation, Yong's equation‐derived corrected MRR was significantly different from those corrected by our equation (3.99 ± 1.51 vs. 4.04 ± 1.53, *p* < 0.001) and also showed a significant difference from true MRR in the validation cohort (3.99 ± 1.51 vs. 4.13 ± 1.71, *p* = 0.046).

### 3.4 True MRR cut‐off values corresponding to CFR, IMR, and RRR cut‐off values

Pre‐PCI true MRR showed significant correlation with CFR (*r* ^2^ = 0.53, *p* < 0.001) and RRR (*r* ^2^ = 0.63, *p* < 0.001), respectively. The best cut‐off values of pre‐PCI true MRR corresponding to CFR = 2.0 and 2.5 were 3.27 (area under the curve [AUC] = 0.86, 95% confidence interval [CI] 0.82–0.90, *p* < 0.001) and 4.08 (AUC = 0.90, 95% CI 0.87–0.93, *p* < 0.001), respectively. There was also a significant correlation between true MRR and IMR, although less robust (*r* ^2^ = 0.10, *p* < 0.001). The best cut‐off values of pre‐PCI true MRR, corresponding to IMR = 25.0 and RRR = 3.5 were 4.61 (AUC = 0.64, 95% CI 0.58–0.70, *p* < 0.001) and 4.08 (AUC = 0.92, 95% CI 0.90–0.95, *p* < 0.001), respectively.

### 3.5 Change in MRR and the relationship between MRR, CFR, and RRR after PCI

Post‐PCI true MRR values significantly decreased (4.14 ± 1.78 vs. 3.70 ± 1.87, *p* < 0.001; Figure 6). Notably, a relatively low agreement was observed between pre‐ and post‐PCI true MRR values when categorized by the best cut‐off value corresponding to CFR values of 2.5 (kappa = 0.238). There remained a significant correlation between post‐PCI true MRR and RRR (*r* ^2^ = 0.97, *p* < 0.001).

**FIGURE 6:** Changes in MRR values after PCI. True MRR significantly decreased after PCI. Abbreviations are shown in Figure 2.

### 3.6 Determinants of the pre‐PCI low true MRR values

Table 2 shows the univariate and multivariate logistic regression analyses to predict the target vessels with pre‐PCI decreased true MRR (MRR < 4.08, threshold corresponding to CFR = 2.5). Pre‐PCI higher IMR and lower CFR were independent predictors of the vessels with decreased pre‐PCI true MRR.

**TABLE 2:** Univariate and multivariate logistic regression analysis for predicting pre‐PCI decreased true MRR (MRR < 4.08).

	Univariate analysis			Multivariate analysis		
	HR	95% CI	*p* value	HR	95% CI	*p* value
Age	1.04	1.02–1.07	<0.001			
Male	0.79	0.44–1.40	0.45			
BMI	0.92	0.87–0.99	0.015			
Hypertension	1.10	0.67–1.80	0.71			
Diabetes Mellitus	1.16	0.76–1.77	0.50			
HbA1c	1.03	0.85–1.25	0.75			
Baseline Hs‐TnI	1.00	1.00–1.00	0.70			
eGFR	1.00	0.99–1.00	0.62			
Log (NT‐pro BNP)	1.20	1.06–1.36	0.005			
LVEF	0.99	0.97–1.01	0.53			
E/e'	1.09	1.03–1.15	0.0014			
Rest P_*d*_/P_*a*_	0.18	0.020–1.69	0.13			
Pre‐PCI FFR	2.70	0.29–25.20	0.38			
Pre‐PCI CFR	0.10	0.063–0.016	<0.001	0.12	0.070–0.19	<0.001
Pre‐PCI IMR	1.04	1.02–1.06	<0.001	1.03	1.00–1.06	0.029
Coronary wedge pressure	0.99	0.96–1.01	0.32			
SYNTAX score	1.02	0.99–1.05	0.26			

Abbreviations: BMI, body mass index; CFR, coronary flow reserve; CI, confidence interval; E/e', early mitral flow velocity to early mitral annular velocity; eGFR, estimated glomerular filtration rate; FFR, fractional flow reserve; HR, hazard ratio; IMR, index of microcirculatory resistance; LVEF, left ventricular ejection fraction; MRR, microvascular resistance reserve; PCI, percutaneous coronary intervention.

## 4 DISCUSSION

In this study, we first sought to derive the equation for estimating FFR_*cor*_ without knowing P_*w*_, as shown in the study by Yong et al. (Yong et al., 2013) in the presence of FFR‐verified functionally significant stenosis for MRR correction. Then, we calculated corrected MRR values using MRR_*app*_ and calculated FFR_*cor*_ values using the derived formula, as suggested by de Bruyne et al. (2021) We validated these corrected MRR values in comparison with true MRR values in the validation cohort. We further evaluated the true pre‐PCI MRR cut‐off values corresponding to reported CFR, IMR, and RRR threshold values in the presence of functionally significant stenosis. We also evaluated the agreement of MRR for the assessment of microvascular dysfunction in comparison with IMR and between pre‐ and post‐PCI MRR values. Finally, the changes in true MRR after uncomplicated PCI were assessed, and predictors of lower pre‐PCI true MRR were explored.

The important findings of this study are as follows; (1) FFR_*cor*_ can be accurately estimated by the equation as follows: FFR_*cor*_ = 1.36 × FFR_*myo*_ – 0.34, showing better performance compared with Yong's formula; (2) in the presence of functionally significant stenosis, corrected MRR can be accurately calculated by the equation as follows: corrected MRR = MRR_*app*_ × (FFR_*myo*_ / FFR_*cor*_) = (MRR_*app*_ × FFR_*myo*_) / (1.36 × FFR_*myo*_ – 0.34); (3) corrected MRR was significantly higher than MRR_*app*_; (4) true MRR cut‐off values in the presence of significant stenosis corresponding to CFR = 2.0 and 2.5 were 3.27 and 4.08, respectively; (5) true MRR cut‐off values corresponding to IMR = 25 was 4.61; (6) true MRR cut‐off value corresponding to RRR = 3.5 was 4.08; (7) true MRR values significantly decreased after PCI and were virtually identical with CFR, while agreement of true MRR before and after PCI was relatively low; (8) pre‐PCI higher IMR values and lower CFR values were independent predictors of low pre‐PCI true MRR.

This is the first study that derived the equation for corrected MRR values in the presence of functionally significant stenosis and validated the equation in the different validation cohort. We also proposed true MRR cut‐off values corresponding to reported CFR, IMR, and RRR cut‐off values, respectively. Furthermore, we presented that the true MRR significantly decreased after uncomplicated PCI, although the agreement between pre‐ and post‐PCI MRR was not high. Recent studies indicate that coronary microvascular dysfunction is a prevalent cause of myocardial ischemia and is associated with poor outcomes. (Fearon et al., 2013; Lee et al., 2016) Microvascular dysfunction is difficult to be visualized and may coexist with obstructive epicardial coronary disease, (Taqueti & Di Carli, 2018; Taqueti et al., 2015) contributing to myocardial ischemia. After successful PCI, preexisting coronary microvascular dysfunction (CMD) or altered microvascular function might emerge and impact the occurrence of ischemic symptoms or adverse events (Misawa et al., 2022; Sechtem et al., 2020; Taqueti et al., 2015) There has been limited data regarding the impact of CMD on prognosis in patients with obstructive epicardial coronary lesions or its behavior after elective PCI. MRR has recently been proposed by Bruyne et al., as defined as the ratio of true resting to hyperemic microvascular resistance. MRR should be corrected in the presence of significant epicardial disease. Our results indicated the wide distribution of MRR and relatively low agreement with IMR before PCI, suggesting that MRR might discriminate the extent of coexisting microvascular dysfunction (MVD) differently from IMR in the presence of significant obstructive disease, although further studies are needed. A strong linear correlation was observed between MRR and CFR. In contrast, a less robust relationship was detected between MRR and IMR, indicating that these two measures for MVD may complementarily provide clinical information about MVD, as suggested above. Further studies are needed to clarify if MRR may provide prognostic information independently of CFR, IMR, or RRR, and whether these indices could be used to discriminate or clarify the relative contribution of myocardial ischemia due to epicardial stenosis and MVD in the presence of significant epicardial disease. Our study provides the clinical characteristics of MRR and true MRR cut‐off values corresponding to CFR, IMR, and RRR cut‐off values to classify the relevance of MVD by these metrics by proposing the reference cut‐off values of each index. Further investigations using these indices for elucidating the clinical significance of CMD in the presence of significant epicardial stenosis were warranted.

## 5 LIMITATIONS

This study was a single‐center retrospective analysis of registered patients' data and pertained to an observational nature; thus, its inherent limitation exists. Rigorous exclusion criteria and the protocol for inclusion limited the number of study patients and may have resulted in a certain level of further selection bias. In the report by Bruyne et al., absolute coronary flow and microvascular resistance measurements were performed using intracoronary continuous saline infusion method for the theoretical framework and MRR validation. In contrast, this study used the thermodilution method (de Bruyne et al., 2021) for CFR and IMR. Currently, both RayFlow® catheter (HEXACATH, Paris, France) and an 0.014” dual pressure and Doppler flow velocity sensor guidewire (ComboWire XT, Philips Volcano) are not commercially available in Japan.

## 6 CONCLUSION

As proposed, without needing P_*w*_ in the presence of significant epicardial stenosis, true MRR can be accurately calculated using calculated FFR_*cor*_ and measured MRR. Pre‐PCI lower CFR and higher IMR were independent predictors of pre‐PCI decreased MRR. Proposed true MRR cut‐off values corresponding to CFR and IMR thresholds representing microvascular dysfunction need to be validated in clinical studies.

## FUNDING INFORMATION

None.

## CONFLICT OF INTEREST STATEMENT

The authors have no conflict of interest to declare.

## ETHICS STATEMENT

Ethical approval was granted by the Tsuchiura Kyodo General Hospital institutional ethics committee (2022FY83) on September 28/2022.
